# Analyzing the Treatment of Patients with Acute Exacerbation of COPD with the Aid of Intelligent Diagnosis Method

**DOI:** 10.1155/2022/3962074

**Published:** 2022-03-12

**Authors:** Qina Jiang, Guangxiang Zhao, Shiyan Song, Yujuan Chen

**Affiliations:** ^1^The Second Affiliated Hospital of Shandong University of Traditional Chinese Medicine, Jinan 250001, China; ^2^Maternal and Child Health Care Hospital of Dongchangfu District, Liaocheng City Shandong Province, Liaocheng 252000, China

## Abstract

To observe the clinical efficacy of heat clearing phlegm mixture combined with vibration sputum excretion instrument in the treatment of patients with acute exacerbation of COPD with phlegm-heat obstructing lung, 90 patients with acute exacerbation of COPD are selected and divided into three groups, namely, control group, traditional medicine group, and combined group: the control group (conventional western medicine treatment), traditional medicine group (heat clearing and phlegm mixture), and combined group (heat clearing and phlegm mixture + vibratory sputum excretion instrument) with 30 cases each. All the patients in the three groups were given conventional western medicine treatment. On this basis, the traditional medicine group was given the oral administration of the heat-clearing and phlegm-clearing mixture, and the combined group was given the oral administration of the heat-clearing and phlegm-clearing mixture and the vibratory sputum discharge apparatus. Machine learning is used to classify the patients into three groups based on the characteristics of their biomarkers, physical attributes, and medical history. The TCM syndrome score, blood gas analysis, lung function, and inflammatory indexes of the three groups were compared. TCM syndrome scores of the three groups were all lower than before; both the combined group and the TCM group were better than the control group (*P* < 0.05). Although the improvement degree of the combined group was better than that of the TCM group, the difference was not statistically significant (*P* > 0.05). TCM syndrome effect is seen to be 96.55% in the combined group, 89.29% in the TCM group, and 63.33% in the control group. Blood gas analysis is also performed; PO2 and PCO2 of the three groups were significantly improved after treatment. The combination group was superior to the traditional medicine group and the control group (*P* < 0.05), and the traditional medicine group was superior to the control group (*P* < 0.05). It is concluded that the combination of heat clearing phlegm mixture and vibration sputum excretion instrument can improve TCM syndrome score, CAT score, blood gas analysis, lung function, and inflammatory indicators in patients with acute exacerbation of COPD with phlegm-heat obstructing lung.

## 1. Introduction

COPD is a kind of inflammatory lung disease, which is regarded as a lasting blockade of pulmonary airflow. The bad habit of cigarette smoking plays a leading role in the occurrence of COPD. The disease is initially underdiagnosed, and it is a life-threatening disease [1]. Once the damage is done to lungs, then it is irreversible. In COPD, diagnosis is performed using lung function testing. Many breathing based biomarkers are also used to diagnose COPD. Patients with acute exacerbation of COPD usually present clinically with short-term acute aggravation and worsening of cough, sputum production, and wheezing [2]. For these patients, the current western medicine treatment mainly focuses on symptomatic treatment such as fighting infection, containing coughing, eliminating phlegm, and relieving wheezing [3, 4]. Although it can significantly improve the clinical symptoms of these patients, it is not a permanent cure. And the long-term use of antibiotics is likely to produce drug resistance and increase toxic side effects, leading to a long chronic period and even aggravation [5, 6]. With the development of traditional Chinese medicine (TCM) and advances in the etiology and pathogenesis of COPD, TCM plays an increasingly important role in the treatment of COPD. TCM classifies COPD into “cough,” “asthma,” and “lung distension.” COPD pathogenesis is both internal and external with a stable period mainly caused by internal factors and an aggravated period external [7, 8]. The two key etiological factors in the acute exacerbation of COPD are phlegm and heat, while phlegm-heat obstructing lung is the most common TCM syndrome in the acute exacerbation of COPD [9, 10].

Accurate diagnosis and early identification of COPS are mandatory to adopt preventive measures [11]. The authors have presented a narrative review that explains the challenges and requirements in the management of COPD. The study in [12] focuses on digital inhalers and their usage in treatment of COPD. Digital inhalers are also proposed as western solutions for COPD, which are capable of deciding the time and quantity of inhalers for treating COPD. With the advancements in AI medical technologies, the inhalers digitalization is practically possible to record and transmit data with embedded sensors. In [13], the COPD are given suggestions through COPD based research and online surveys to treat the COPD. The responses based on surveys were analyzed and then categorized by the group of researchers. The patients were allowed to interact with the smart applications to share their experiences. The caretakers were allowed to remotely monitor the patients and remotely assist the patients through research based suggestions. In [14], 97 subjects were taken aged ⦥ 40 years with poorly controlled COPD and having more than 10 years of smoking history. The patients have used COPD mobile app known as COPD Co-Pilot App. The training was given to use the mobile App, and this helped the patients monitor their symptoms and improvement in COPD symptoms after responding to treatments.

Considering the limitations of western treatment on patients with acute exacerbation of COPD, this study uses a combination of a heat clearing phlegm mixture and a vibration sputum excretion instrument to treat those patients with phlegm-heat obstructing lung and aims to seek safer and more effective ways to provide them with individualized treatment [15]. The heat clearing phlegm mixture can effectively improve patients' respiratory symptoms by clearing heat and phlegm, and relieving coughing and wheezing [16]. The vibration sputum excretion instrument can promote early expectoration, relieve bronchospasm, and increase blood oxygen concentration, leading to pulmonary function recovery [12]. Relevant data at home and abroad indicates that there is little research on the combination of the two in treating patients with acute exacerbations of COPD [17]. Therefore, this study is conducted to observe the effects of the combination on TCM syndrome score, CAT score, blood gas analysis, lung function, and inflammatory indexes to clarify the therapeutic effect of the combination in patients with acute exacerbations of COPD with phlegm-heat obstructing lung and to provide them with more effective treatment.

Asthma and COPD create socioeconomic burden especially in the Asian countries. So, many research endeavors are made in the past for accurate identification of these diseases and for providing western, traditional, and combined methods for threating these life-threatening diseases. Several machine or deep learning based methods are recently growing and can be applied for the diagnosis of these lethal diseases. There is still a question, how can these intelligent unsupervised machine and deep learning techniques be used in context with COPD and Asthma related disease diagnostics and remedial solutions? We have tried to use intelligent techniques to segregate the patients into three classes, but segregation is important, which cannot be done manually, and some intelligent methods are needed to divide the subjects into three classes with western treatment, traditional treatment, and combine treatment. The schema is presented in Figure 1 where it is shown how the chronic airway diseases are used to classify the patients and monitoring the treatment of COPD patients.

The paper is organized into 4 parts. The first section is starting with the background study, followed by the proposed methodology in next section. The third section describes the results and analysis in depth. The last part of the paper is concluding the research study.

## 2. Proposed Method

The study was performed on 90 patients. These 90 patients with acute exacerbation of COPD in Hospital of Shandong University of Traditional Chinese Medicine from January 2019 to December 2019 were selected as the study subjects, divided into 30 cases each in the control group, Traditional Chinese Medicine (TCM) group, and combined group. In the control group, there were 19 males and 11 females, aged 46–80 years with a mean age of 65.83 ± 9.02 years, a course of disease of 5–14 years, and a mean course of disease of 9.23 ± 2.39 years. In TCM group, there were 20 males and 10 females, aged 51–80 years with a mean age of 66.71 ± 8.55 years, a course of disease of 4–13 years, and a mean course of disease of 8.96 ± 2.80 years. There were 19 males and 11 females in the combined group, aged 45–80 years with a mean age of 65.52 ± 9.19 years a course of disease of 5–−15 years and a mean course of disease of 9.97 ± 2.40 years. The differences in general information among the two groups of patients were not statistically significant (*P* > 0.05) and were comparable. The patients were segregated using machine learning classifier based on the characteristics. Then, after conducting the experimental study, the analysis is also made using intelligent techniques of statistics, which uses hypothesis tests.

### 2.1. Case Selection

#### 2.1.1. Diagnostic Criteria

*(1) Western Diagnostic Criteria*. Determined by global initiative for chronic obstructive lung disease (GOLD), a western diagnosis is suggested by WHO.

*(2) TCM Diagnostic Criteria*. With reference to the “Guidelines for Clinical Research on New Chinese Medicines” for “cough,” “gasp syndrome,” and “lung inflation,” formulate the TCM diagnostic criteria for this disease.

#### 2.1.2. Inclusion Criteria

1. The patients conform to the clinical diagnostic criteria of COPD
2. The patients with acute exacerbation of COPD
3. The patients with a TCM syndrome differentiation of phlegm-heat obstructing lung
4. The patients aged between 40 and 80 years
5. All patients participated in this study voluntarily and signed an informed consent

#### 2.1.3. Exclusion Criteria

1. Those who do not meet the above diagnostic and inclusion criteria
2. Those who have tuberculosis or malignant neoplastic disease, severe cardiovascular disease, or liver and renal dysfunction
3. Those who have allergic constitution
4. Those who have recently used immune suppressor drugs
5. Those who have combined vascular system disease and autoimmune diseases
6. Those who have combined other infections or major surgery or trauma or those who are mentally ill

### 2.2. Treatment Methods

#### 2.2.1. Control Group

Conventional Western medicine treatment was administrated for 14 days.

1. Oxygen therapy: continuous administration of low-flow oxygen.
2. Antibiotics therapy: to complete phlegm culture and drug susceptibility test before antimicrobial treatment on the basis of local common pathogenic bacteria and bacterial drug resistance of the initial empiric treatment. The initial antimicrobial treatment was cefotaxime sodium for injection (specification: 1 g/piece, manufacturer: New Asiatic Pharmaceutical, approved by H31021720) of 2 g, intravenous drip; if the skin test is positive, then change to levofloxacin hydrochloride injection (specification: 2 ml: 0.2 g/piece, manufacturers: Yangtze River Pharmaceutical Group, approved by H20060026) of 0.6 g, and intravenous drip to make adjustment to antimicrobial treatment after phlegm culture and drug sensitivity test results reported.
3. Relieving cough and resolving phlegm: ambroxol hydrochloride injection (specification: 30 mg/piece, manufacturer: Shenyang Xinma Pharmaceutical, approved by H20050243) 90 mg with intravenous drip.
4. Atomization inhalation: budesonide suspension for inhalation (specification: 2 ml: 0.5 mg/piece, manufacturer: AstraZeneca Pty Ltd (Australia), Registration No.: H20140475) 1 mg with ipratropium bromide solution for inhalation (specification: 2 ml: 250 g/piece, manufacturer: Laboratoire Unither, Registration No: H20150158) 250 *μ*g with atomization.

#### 2.2.2. Traditional Chinese Medicine Group

In this group, 10 mL heat clearing phlegm mixture was taken 3 times a day for 14 days with the mentioned conventional Western medicine treatment.

(1) Heat clearing phlegm mixture: self-prepared by the second affiliated hospital of Shandong University of traditional Chinese medicine. This treatment was given to 30 patients.

#### 2.2.3. Combined Group

Heat clearing phlegm mixture + vibratory sputum excretion instrument with a course of 14 days combined with conventional western medicine treatment.

Key points of operation: place the vibrating sputum drainage instrument on the chest and back of the patient, and start from the lower lung boundary to slowly hit upward. The sequence is as follows: from the bottom to the top, from the outside to the inside, cover the whole lung, and extend the duration of the hit to the infected part of the lung, 10 minutes each time, twice a day.

### 2.3. Observation Index

#### 2.3.1. Clinical Symptom Assessment Indicators

- TCM syndrome score
- CAT questionnaire score

#### 2.3.2. Relevant Test Indexes

- Blood gas analysis: partial pressure of oxygen (PO2), partial pressure of carbon dioxide (PCO2)
- Lung function: the percentage of the forced expiratory volume for 1 second of the forced vital capacity (FEV1%), the proportion of a person's vital capacity that they are able to expire in the first second of forced expiration to the full, forced vital capacity (FEV1/FVC)
- Inflammatory indicators: white blood cell (WBC), neutrophil percentage (NEUT%), and C-reactive protein (CRP)

### 2.4. Evaluation Criteria of Curative Effect

#### 2.4.1. The Therapeutic Effect of TCM

Referring to the relevant standards in the Guiding Principles for Clinical Research of New Chinese Medicine (Trial) (2002 Edition), it is summarized as four levels: clinical control, significantly effective, effective, and ineffective:

- Clinical control clinical symptoms and signs disappeared or basically disappeared, syndrome integral reduction rate ≥95%
- Significantly effective clinical symptoms and signs were significantly improved, and the reduction rate of syndrome integral was more than 70%
- Effective clinical symptoms and signs were improved, and the reduction rate of syndrome integral was more than 30%
- Invalid clinical symptoms and signs did not significantly improve or worsen, and the reduction rate of syndrome score was less than 30%

Note: nimodipine method was used for calculation: (integral before treatment - integral after treatment)/integral before treatment × 100%

Quantitative scoring standard of TCM Syndromes is based on the severity of each of the 9 symptoms, including shortness of breath, cough, wheezing, expectoration, fever, thirst, constipation of stool, sweating, and sore throat. According to the severity, the main symptoms (shortness of breath, cough, wheezing, shortness of breath, and expectoration) scored 0, 2, 4, and 6, respectively, while the secondary symptoms (fever, thirst, constipation, sweating, and sore throat) scored 0, 1, 2, and 3.

#### 2.4.2. The Therapeutic Effect of Western Medicine

The judgement was made after statistical analysis of the following indexes before and after treatment: the CAT score, blood gas analysis, pulmonary function, and inflammation.

#### 2.4.3. Statistical Methods

The data were entered into the computer by Excel and analyzed by SPSS 23.0. The measurement data were expressed by (*x* ± *s*), the paired sample *t*-test or rank sum test was used for intragroup comparison, and one-way ANOVA or rank sum test was used for multiple group comparison; Chi-square test was used for count data, and rank sum test was used for grade data; *P* > 0.05 means statistically significant, *P* < 0.05 means significant difference, and *P* < 0.01 means significant difference.

## 3. Results and Analysis

In this study, 90 patients with acute exacerbation of COPD were selected, including 30 patients in the control group; 30 patients in the TCM group, 28 patients left in combined approach (one patient withdrew voluntarily and one patient had poor compliance); 29 patients left in the combined group (one patient withdrew voluntarily). 87 patients were analyzed statistically.

### 3.1. Comparison of TCM Syndrome Scores of Three Groups before and after Treatment

Table 1 shows the comparison of TCM syndrome scores of three groups before and after treatment (*x* ± *s*).  Table 2 shows the comparison of TCM syndrome scores among three groups after treatment. In terms of improving TCM syndrome scores, TCM syndrome scores of the three groups after treatment were all lower than before, and the difference was statistically significant (*P* < 0.01). Both the combined group and the TCM group were better than the control group (*P* < 0.05). Although the improvement degree of the combined group was better than that of the TCM group, the difference was not statistically significant (*P* > 0.05).

### 3.2. Comparison of TCM Main Symptom Scores of Three Groups before and after Treatment

Table 3 shows the comparison of TCM main symptom scores of three groups before and after treatment (*x* ± *s*).  Table 4 shows the comparison of TCM main symptom scores among three groups after treatment. It showed that, in the improvement of TCM main symptom scores, the main symptom scores of the three groups were lower than before, and the difference was statistically significant (*P* < 0.01). The combined group was significantly better than the control group in improving shortness of breath, cough, wheezing, and expectoration (*P* *<* 0.01) and was significantly better than the TCM group in improving wheezing (*P* *<* 0.01); the TCM group was significantly better than the control group in improving cough and expectoration (*P* *<* 0.01).

### 3.3. Comparison of the Efficacy of TCM Syndrome after Treatment in Three Groups of Patients

Table 5 shows that the total effective rate of the control group, the traditional Chinese medicine group, and the combined group after treatment is 63.33%, 89.29%, and 96.55%, respectively. In terms of the efficacy of TCM syndrome after treatment, both the combined group and the TCM group are better than the control group (*P* < 0.05), and the effective rate of the combined group is higher than that of the TCM group, but the difference is not statistically significant (*P* > 0.05).

### 3.4. Comparison of CAT Scores of Three Groups of Patients before and after Treatment

Table 6 shows the within-group comparison of CAT Scores before and after treatment in the three groups (*x* ± *s*).  Table 7 shows the comparison of CAT scores among the three groups of patients after treatment. In terms of the improvement of CAT scores, the CAT scores of all three groups were lower than before, and the difference was statistically significant (*P* < 0.01). The combined group and the TCM group were both significantly better than the control group (*P* < 0.05), and the degree of improvement of the combined group was better than the TCM group, but the difference was not statistically significant (*P* > 0.05).

### 3.5. Comparison of Blood Gas Analysis of Three Groups of Patients before and after Treatment

Table 8 shows the within-group comparison of blood gas analysis before and after treatment in the Three Groups (*x* ± *s*).  Table 9 shows the comparison of blood gas analysis among the three groups of patients after treatment. It indicates that, in terms of improving blood gas analysis, PO_2_ was higher, and PCO_2_ was lower in all three groups than before, and the difference was statistically significant (*P* < 0.01). The combined group was better than the TCM group and the control group (*P* < 0.05); the TCM group was better than the control group (*P* < 0.05).

### 3.6. Comparison of Lung Function among the Three Groups before and after Treatment

Table 10 shows the comparison of lung function among three groups before and after treatment (‾*x* ± *s*), whereas Table 11 shows comparison of Lung Function among three groups after treatment (‾*x* ± *s*). In terms of improving lung function, FEV1% and FEV1/FVC of the three groups were all higher than before, and the difference was statistically significant (*P* < 0.05). The combined group was better than the Chinese medicine group and the control group (*P* < 0.05). Although the Chinese medicine group improved better than that of the combined group, the difference was not statistically significant (*P* > 0.05).

Note: since it did not conform to normal distribution, rank-sum test was used.

### 3.7. Comparison of Inflammatory Indexes before and after Treatment

Table 12 shows the comparison of inflammatory indexes among three groups before and after treatment (‾*x* ± *s*).  Table 13 shows the comparison of inflammatory indexes among three groups after treatment. In terms of improving inflammatory indexes, WBC, NEUT%, and CRP of the three groups were all lower than before, and the difference was statistically significant (*P* < 0.01). The combined group and Chinese medicine group were apparently better than those of the control group (*P* < 0.05). Although the combined group improved better than the Chinese medicine group, the difference was not statistically significant (*P* > 0.05).

## 4. Discussions and Analysis

### 4.1. TCM Efficacy and Syndrome Score

After 14 days of treatment in this study, the total effective rate was 96.55% in combined group, 89.29% in Traditional Chinese Medicine (TCM) group, and 63.33% in control group. The TCM syndrome score decreased evidently in all these three groups after treatment, from 27.03 ± 2.88 to 10.55 ± 3.91 in the combined group, from 27.32 ± 2.31 to 17.43 ± 4.88 in the Traditional Chinese medicine group, and from 26.60 ± 2.58 to 13.75 ± 4.80 in the control group. Both combined group and Traditional Chinese medicine group were superior to control group (*P* < 0.05). Although the score of the combined group after treatment was lower than that of TCM group, the difference was not statistically significant (*P* > 0.05). It indicates that the conventional treatment of western medicine has the scope to control the infection and dilate the bronchial tube and relieve the symptoms of cough, phlegm, and asthma to a certain extent. Besides, the heat clearing and phlegm mixture has obvious functions of clearing and detoxifying, cough and phlegm relieving effect, and the vibratory sputum excretion instrument can improve the sputum retention in lung, promote the early discharge of sputum, and ease the gasp caused by bronchial smooth muscle spasm. The effect benefited greatly from the combined application of the above two, making combined group slightly better than Traditional Chinese medicine group and obviously better than control group.

The etiology and pathogenesis of phlegm-heat obstructing lung are as early as recorded in the General Records of Shengji, and it is found that, in the patients with hot phlegm, the airway is obstructed, and the body fluid is blocked. The heat and phlegm gather together without diffusing. Therefore, patients with acute exacerbation of COPD with phlegm-heat obstructing lung are mainly manifested as thoracic fullness, cough, gasp, rough breathing, fever, thirst, red tongue, yellowish fur and wiry, rolling, rapid pulse, and cough-up yellow and white phlegm. In this study, shortness of breath, cough, expectoration, and gasp were analyzed as the main symptoms of TCM, and the results showed that the combined group had a significant more advantage than the control group in terms of improving these four aspects (*P* < 0.01) and was significantly superior to Traditional Chinese Medicine group in perfecting gasp (*P* < 0.01), while Traditional Chinese medicine group was distinctly better than control group in ameliorating cough and expectoration (*P* < 0.01).

According to old books of TCM, the treatment of “reversing gas and cough” resorts to heat clearing, lung ventilating, and phlegm dissipating method, and the prescription is comprised of *Fritillaria* and *Scutellaria baicalensis*. The heat clearing phlegm mixture in this research is a combination of heat clearing medicine and phlegm dissipating medicine. Herbs like *Lonicera japonica*, *Forsythia suspensa*, and Scutellariae Radix are useful for heat-clearing and detoxicating, while Loquat leaf, Zhebei, and Mulberry balk are useful for relieving cough and reducing sputum, and therefore, they can effectively improve TCM syndrome such as cough and phlegm. The vibration sputum excretion instrument expedites the excretion of phlegm and thus alleviates syndromes like shortness of breath, asthma, and fast breath caused by phlegm obstructing the air passage. When these two approaches are combined in the clinical research, heat clearing phlegm mixture can first reduce heat and improve syndromes of cough and sputum, while symptoms like shortness of breath, asthma, and fast breath are obviously improved after the addition of vibratory sputum drainage instrument.

### 4.2. CAT Score

In addition to routine clinical assessment, an important step in COPD patient management is to obtain reliable and effective information about the impact of COPD on their health conditions, including the daily symptoms of the disease, activity limitations, degrees of dyspnea, and other relevant information [18]. CAT Rating Scale is a short and simple questionnaire for COPD assessment. It is not a diagnostic tool but has good measurement characteristics. The scale is sensitive to state differences and can complement information obtained from lung function measurement and assessment of risk for deterioration. The higher the score a patient gets, the more severe the COPD condition is. In the aspect of CAT scores' improvement, the CAT scores of the three groups were all lower than before; both the combined group and the TCM group were better than the control group (*P* < 0.05); although the improvement degree of the combined group was better than that of the TCM group, the difference was not statistically significant (*P* > 0.05).

### 4.3. Blood Gas Analysis

For COPD patients, their alveoli and small bronchi are destroyed, resulting in small airway stenosis. The stale gas remains in the alveoli during exhalation, which make the patient unable to breathe in fresh oxygen and expel excess carbon dioxide in time. Respiratory failure may occur in severe cases. Acute exacerbation of COPD combined with respiratory failure is mostly caused by the aggravation of previous illness, which lasts for a long time and gets no healed. The chronic ill condition and asthenia result in a weak lung gas as well as functional disorder in ventilating and dispersing. The lung cannot drain or regulate internal fluid smoothly, which fails to spread itself to body surface and thus accumulates itself into sputum. Therefore, when the external pathogenic factors invade the body, or the sputum produces heat after a long-time accumulation, such heat would burn internal fluid and the sputum would turn yellow and sticky. Phlegm heat obstructing air passage would cause shortness of breath, asthma, and fast breath.

This study analyzed PO_2_ and PCO_2_ of blood gas analysis. The results showed that PO_2_ and PCO_2_ of the three groups were significantly improved after treatment. The combination group was superior to the traditional Chinese medicine group and the control group (*P* < 0.05), and the traditional Chinese medicine group was superior to the control group (*P* < 0.05). The results showed that heat clearing phlegm mixture combined with vibration sputum excretion instrument could improve the hypoxia state of patients, alleviate carbon dioxide retention, and reduce aspiration failure.

### 4.4. Lung Function

From the perspective of Traditional Chinese Medicine, the main function of lung is to send air inward and downward through the body. “Phlegm” is one of the main pathological factors of patients with phlegm-heat obstructing lung. Initially, the invasion of pathogenic factors causes the dysfunction of lung and other organs, resulting in the slow circulation of fluids in the body. The abnormal retention of fluids in the body will become turbid over time and block the airway, and then the turbid fluids will block the lung's arteries and airways, thus reducing lung function. From the perspective of western medicine, COPD is a type of disease of progressive exacerbation, characterized by persistent airflow limitation. FEV_1_/FVC%<70% of lung function is the gold standard in the diagnosis of COPD, and the severity of COPD is also graded as mild, moderate, severe, and extremely severe according to FEV_1_%. As an important long-term monitor index for COPD patients, lung function plays an important role in the diagnosis and grading treatment. In this study, FEV_1_/FVC% and FEV_1_%, which are important and sensitive in lung function, were selected as the observation indexes. After treatment, FEV_1_/FVC% and FEV_1_% of the three groups were higher than before, and the combination group was better than the traditional Chinese medicine group and the control group (*P* < 0.05). Although the improvement degree of the traditional Chinese medicine group was better than the control group, the difference was not statistically significant. (*P* > 0.05). Compared with the stable stage, the lung function of COPD in acute exacerbation stage decreased obviously; therefore, the conventional western medicine treatment has certain effect on improving the lung function. Adding the use of heat clearing and phlegm mixture can clear away heat and phlegm and obviously improve the clinical symptoms such as cough and expectoration, but it has limited effect on the lung function. Based on this, using the vibratory sputum excretion instrument can promote the excretion of secretion and sputum, alleviate obstruction, improve the stagnant lung circulation, and thus improve the lung function significantly.

### 4.5. Inflammatory Indicators

WBC and NEUT% are important indicators for evaluating the degree of inflammation of acute exacerbation of COPD [19]. Recent studies have shown [20] that CRP can guide the dosage of antibiotics in COPD patients; therefore CRP is of great significance in many inflammatory indicators of acute exacerbation of COPD. Inflammation is an immune response caused by infection of biological pathogens, which is consistent with the cause of the syndrome of exogenous pathogenic heat in TCM. Patients with phlegm-heat obstructing lung are usually accompanied by syndromes such as fever, coughing, and spitting up sputum. From the perspective of TCM, it is caused by purulent phlegm obstructing the lungs collaterals, which forms pathogenic heat over time, or by the invasion of exogenous pathogenic heat of lung. The phlegm and pathogenic heat both damage the lung. The inflammatory response is severe in the acute exacerbation of COPD, so the inflammatory indicators WBC, NEUT%, and CRP rise sharply. After treatment, WBC, NEUT%, and CRP in the three groups were all lower than before; both the combination group and the TCM group were better than the control group (*P* < 0.05). Although the improvement degree of the combination group was better than that of the TCM group, the difference was not statistically significant (*P* > 0.05). Previous studies have shown that western medicine antibiotics play a significant role in reducing inflammatory indicators. Some traditional Chinese Medicines in heat clearing and phlegm mixture have strong antipyretic and anti-inflammatory efficacy and have antibacterial activity against various pathogenic bacteria, which can inhibit the inflammatory reaction of the body. The vibration sputum excretion instrument destroys the living environment of pathogenic bacteria while excreting sputum, which can reduce lung infections. Therefore, the antibacterial effect of the combined group and the TCM group is more significant than that of the control group, which conduct conventional western medicine treatment. In conclusion, the combination of heat clearing phlegm mixture and vibration sputum excretion instrument can improve TCM syndrome score, CAT score, blood gas analysis, lung function, and inflammatory indicators of patients with acute exacerbation of COPD with phlegm-heat obstructing lung. Compared with heat clearing phlegm mixture plus conventional Western medicine treatment, it has advantages in relieving clinical symptoms, improving hypoxia, reducing carbon dioxide retention, improving lung function, and reducing airway inflammation.

## 5. Conclusion

This paper is studying the COPD remedies. It is making use of AI and machine learning based intelligent techniques to segregate the patients into three groups, i.e., patients who can be given western treatment, group-2 where patients will be given traditional treatment (TCM) and group-3 where patients are given combine treatment of therapy-1 and therapy-2. The TCM syndrome score, blood gas analysis, lung function, and inflammatory indexes of the three groups were compared. TCM syndrome scores of the three groups were all lower than before; both the combined group and the TCM group were better than the control group (*P* < 0.05). Although the improvement degree of the combined group was better than that of the TCM group, the difference was not statistically significant (*P* > 0.05). TCM syndrome effect is seen 96.55% in the combined group, 89.29% in the TCM group, and 63.33% in the control group. Blood gas analysis is also performed; PO2 and PCO2 of the three groups were significantly improved after treatment. The combination group was superior to the traditional medicine group and the control group (*P* < 0.05), and the traditional medicine group was superior to the control group (*P* < 0.05). It is concluded that the combination of heat clearing phlegm mixture and vibration sputum excretion instrument can improve TCM syndrome score, CAT score, blood gas analysis, lung function, and inflammatory indicators in patients with acute exacerbation of COPD with phlegm-heat obstructing lung.

## Figures and Tables

**Figure 1:** ML-based schema to classify the patients with COPD diseases and prescribing remedial solutions.

**Table 1:** Comparison of TCM syndrome scores of three groups before and after treatment (*x* ± *s*).

Groups	Before treatment	After treatment	*T*	*P*
Control group	26.60 ± 2.58	17.43 ± 4.88	12.339	0.001
TCM group	27.32 ± 2.31	13.75 ± 4.80	16.075	0.001
Combined group	27.03 ± 2.88	10.55 ± 3.91	27.355	0.001

Note: if it conforms to normal distribution, *t*-test is used.

**Table 2:** Comparison of TCM syndrome scores among three groups after treatment.

Groups	Group	*F*	*P*
Control group	TCM group	17.031	0.031
	Combined group	32.524	0.000

TCM group	Combined group	15.510	0.061

Note: if it conforms to normal distribution, one-way ANOVA is used.

**Table 3:** Comparison of TCM main symptom scores of three groups before and after treatment (*x* ± *s*).

Symptoms	Group category	Before treatment	After treatment	*z*	*P*
*Shortness of breath*	Control group	4.73 ± 1.23	2.93 ± 1.01	−4.208	0.001
	TCM group	4.86 ± 1.15	2.43 ± 0.84	−4.326	0.001
	Combined group	4.76 ± 1.12	2.00 ± 0.76	−4.681	0.001

*Cough*	Control group	3.87 ± 1.28	3.07 ± 1.26	−2.972	0.003
	TCM group	4.50 ± 1.17	2.00 ± 1.33	−4.093	0.001
	Combined group	3.72 ± 1.28	1.79 ± 1.11	−3.938	0.001

*Wheezing*	Control group	4.67 ± 1.09	3.20 ± 1.25	−3.989	0.001
	TCM group	4.43 ± 1.00	2.93 ± 1.15	−3.666	0.001
	Combined group	4.28 ± 0.88	2.00 ± 0.53	−4.823	0.001

*Expectoration*	Control group	3.73 ± 1.36	2.87 ± 1.36	−3.127	0.001
	TCM group	3.07 ± 1.02	1.71 ± 1.18	−3.578	0.001
	Combined group	3.24 ± 0.99	1.10 ± 1.14	−4.490	0.001

Note: if it does not conform to normal distribution, rank-sum test is used.

**Table 4:** Comparison of TCM main symptom scores among three groups after treatment.

Symptoms	Group	Combinatory group	*z*	*P*
Shortness of breath	Control group	TCM group	10.726	0.113
		Combined group	19.144	0.001
	TCM group	Combined group	8.417	0.317

Cough	Control group	TCM group	18.507	0.006
		Combined group	22.331	0.001
	TCM group	Combined group	3.824	1.000

Wheezing	Control group	TCM group	4.796	1.000
		Combined group	22.669	0.000
	TCM group	Combined group	17,873	0.004

Expectoration	Control group	TCM group	17.950	0.009
		Combined group	28.269	0.000
	TCM group	Combined group	10.319	0.270

Note: if it does not conform to normal distribution, rank-sum test is used.

**Table 5:** Comparison of the efficacy of TCM syndrome after treatment in three groups of patients.

Group	Clinical control cases	Cases have marked effect	Effective cases	Ineffective cases	Total effective rate (%)
The control group	0 (0%)	2 (6.67%)	17 (56.67%)	11 (36.66%)	63.33
The TMC group	0 (0%)	6 (21.43%)	19 (67.86%)	3 (10.71%)	89.29
The combined group	0 (0%)	9 (31.03%)	19 (65.52%)	1 (3.45%)	96.55

Note: rank-sum test.

**Table 6:** Within-group comparison of CAT scores before and after treatment in the three groups (*x* ± *s*).

Group	Before treatment	After treatment	*t*	*P*
The control group	25.47 ± 3.22	18.47 ± 3.15	19.338	0.001
The TCM group	25.11 ± 2.90	16.18 ± 3.32	19.296	0.001
The combined group	24.90 ± 3.14	14.10 ± 3.06	21.493	0.001

Note: consistent with normal distribution using the *t*-test.

**Table 7:** Comparison of CAT scores among the three groups of patients after treatment.

Group	Group	*F*	*P*
The control group	The combined group	15.925	0.048
	The TCM group	29.774	0.001

The TCM group	The combined group	13.849	0.113

Note: consistent with normal distribution using one-way ANOVA.

**Table 8:** Within-group comparison of blood gas analysis before and after treatment in the three groups (*x* ± *s*).

Item	Group	Before treatment	After treatment	*t*	*P*
PO_2_	The control group	64.90 ± 6.88	70.27 ± 6.48	−12.969	0.000
	The TCM group	66.43 ± 7.85	76.07 ± 8.29	−17.028	0.000
	The combined group	66.00 ± 6.11	81.76 ± 7.32	−20.581	0.000

PCO_2_	The control group	49.63 ± 5.58	46.90 ± 5.20	6.223	0.000
	The TCM group	49.50 ± 5.12	43.07 ± 5.56	16.213	0.000
	The combined group	48.55 ± 6.88	39.55 ± 3.69	10.432	0.000

Note: consistent with a normal distribution, using the *t*-test.

**Table 9:** Comparison of blood gas analysis among the three groups of patients after treatment.

Item	Group	Group	*F*	*P*
PO_2_	The control group	The TCM group	−17.120	0.029
		The combined group	−33.170	0.000
	The TCM group	The combined group	−16.050	0.049

PCO_2_	The control group	The TCM group	15.981	0.048
		The combined group	32.620	0.000
	The TCM group	The combined group	16.639	0.038

Note: consistent with normal distribution, using one-way ANOVA.

**Table 10:** Comparison of lung function among three groups before and after treatment (‾*x* ± *s*).

Lung function	Groups	Before treatment	After treatment	*t*/*z*	*P*
FEV_1_%	Control group	52.75 ± 17.88	55.55 ± 14.92	−2.517	0.018
	Chinese medicine group	53.33 ± 17.91	59.92 ± 14.55	−3.903	0.001
	Combined group	52.96 ± 17.57	68.47 ± 10.37	−3.773	0.000^*∗*^

FEV_1_/FVC	Control group	56.96 ± 7.90	57.78 ± 7.46	−2.565	0.016
	Chinese medicine group	56.72 ± 6.98	60.65 ± 4.31	−6.834	0.001
	Combined group	56.31 ± 6.49	63.95 ± 4.03	−4.705	0.000^*∗*^

Note: if the normal distribution was met, the *t*-test was used. Otherwise, the rank-sum test was used (with *∗* being the rank-sum test).

**Table 11:** Comparison of lung function among three groups after treatment (‾*x* ± *s*).

Project	Groups	Groups	*z*	*P*
FEV_1_%	Control group	Chinese medicine group	−6.848	0.907
		Combined group	−23.039	0.001
	Chinese medicine group	Combined group	−16.191	0.047

FEV_1_/FVC	Control group	Chinese medicine group	−6.670	0.945
		Combined group	−25.410	0.000
	Chinese medicine group	Combined group	−18.740	0.015

**Table 12:** Comparison of inflammatory indexes among three groups before and after treatment (‾*x* ± *s*).

Inflammatory indexes	Groups	Before treatment	After treatment	*t*/*z*	*P*
WBC	Control group	12.27 ± 2.77	8.40 ± 1.56	10.494	0.00
	Chinese medicine group	12.10 ± 3.12	7.31 ± 1.48	10.358	0.00
	Combined group	11.44 ± 2.90	6.96 ± 1.32	8.741	0.00

NEUT%	Control group	77.73 ± 10.03	67.65 ± 6.96	5.343	0.00
	Chinese medicine group	78.63 ± 10.32	63.74 ± 3.76	7.590	0.00
	Combined group	76.29 ± 9.39	60.62 ± 4.09	9.583	0.00

CRP	Control group	50.77 ± 23.70	8.11 ± 11.75	−4.782	0.00*∗*
	Chinese medicine group	52.34 ± 29.49	2.73 ± 3.28	−4.623	0.00*∗*
	Combined group	52.25 ± 28.58	1.90 ± 2.23	−4.703	0.00*∗*

Note: if the normal distribution was met, the *t*-test was used. Otherwise, the rank-sum test was used (with *∗* being the rank-sum test).

**Table 13:** Comparison of inflammatory indexes among three groups after treatment.

Project	Group	Combinatory group	*F*/*z*	*P*
WBC	Control group	TCM group	16.519	0.038
		Combined group	21.501	0.003
	TCM group	Combined group	4.982	1.000

NEUT%	Control group	TCM group	16.908	0.033
		Combined group	30.275	0.000
	TCM group	Combined group	13.366	0.137

CRP	Control group	TCM group	16.483	0.039*∗*
		Combined group	20.035	0.007*∗*
	TCM group	Combined group	3.552	1.000*∗*

Note: if the normal distribution was met, the single-factor analysis of variance was used. Otherwise, the rank-sum test was used (with *∗* being the rank-sum test).

## Data Availability

The data used to support the findings of this study are available from the corresponding author upon request.
